# Empirical Modeling of Physiochemical Immune Response of Multilayer Zinc Oxide Nanomaterials under UV Exposure to Melanoma and Foreskin Fibroblasts

This article has been retracted.

**DOI:** 10.1038/srep46603

**Published:** 2017-04-24

**Authors:** Muhammad Fakhar-e-Alam, M. Waseem Akram, Seemab Iqbal, K. S. Alimgeer, M. Atif, K. Sultana, M. Willander, Zhiming M. Wang

**Affiliations:** 1 Institute of Fundamental and Frontier Science, University of Electronic Science and Technology of China, 610054 Chengdu, China; 2 Department of Science and Technology, Campus Norrköping, Linköping University, SE-601 74 Norrköping, Sweden; 3 Department of Physics, GC University, 38000 Faisalabad, Pakistan; 4 COMSATS Institute of Information Technology, Islamabad, Pakistan; 5 Department of Physics and Astronomy, College of Science, King Saud University, Riyadh, Saudi Arabia; 6 National Institute of Laser and Optronics, Nilore, Islamabad, Pakistan

## Abstract

Carcinogenesis is a complex molecular process starting with genetic and epigenetic alterations, mutation stimulation, and DNA modification, which leads to proteomic adaptation ending with an uncontrolled proliferation mechanism. The current research focused on the empirical modelling of the physiological response of human melanoma cells (FM55P) and human foreskin fibroblasts cells (AG01518) to the multilayer zinc oxide (ZnO) nanomaterials under UV-A exposure. To validate this experimental scheme, multilayer ZnO nanomaterials were grown on a femtotip silver capillary and conjugated with protoporphyrin IX (PpIX). Furthermore, PpIX-conjugated ZnO nanomaterials grown on the probe were inserted into human melanoma (FM55P) and foreskin fibroblasts cells (AG01518) under UV-A light exposure. Interestingly, significant cell necrosis was observed because of a loss in mitochondrial membrane potential just after insertion of the femtotip tool. Intense reactive oxygen species (ROS) fluorescence was observed after exposure to the ZnO NWs conjugated with PpIX femtotip model under UV exposure. Results were verified by applying several experimental techniques, e.g., ROS detection, MTT assay, and fluorescence spectroscopy. The present work reports experimental modelling of cell necrosis in normal human skin as well as a cancerous tissue. These obtained results pave the way for a more rational strategy for biomedical and clinical applications.

Zinc oxide is a promising material because of its novel applications in the fields of basic and applied science. ZnO itself and with PpIX has gained popularity in the field of medical science. In this modern age, very efficient and quick response treatment modalities are a basic need. Bio-nanotechnology is an emerging field because of its diverse applications. The propensity for accumulation in tissue is an obstacle to current research. Nanoparticles drug delivery is currently a hot topic; there are significant challenges for pharmacists and oncologists to overcome in regards to the deficiency in drug bioavailability. More sophisticated, stable, and adequate treatment techniques are needed. Scientists have been working towards improving drug uptake in targeted sites for the treatment of severe diseases of malignancy/premalignancy in the last three decades. Affected patients are still waiting for a big breakthrough with an efficacious response. Nano-technological-based treatment modalities are limited on the basic level because of a lack of efficacy and clinical safety protocols. Photodynamic therapy (PDT) is a non-invasive treatment modality based on the pharmacokinetics of drugs both individually and as nanomaterial hybrids in malignant cells under exposure to suitable wavelengths of light. The excited photosensitizer transfers its energy to molecular oxygen, which permits the photosensitizer to settle down to its ground state and to excite the molecular state of oxygen (triplet oxygen) into a singlet excited state. Singlet oxygen is extremely responsive to biomolecules and has effective results especially in cancerous cells via production of reactive oxygen species which tend to promote apoptosis or necrosis^1^. The necrotic effect of PDT *in vivo* is based on preferential retaining of the photosensitizer within tumorous parts of tissue followed by a controlled luminance target site. Two principal mechanisms can be considered for PDT-mediated tumour eradication, namely, direct damage to the tumour cells and stroma. The latter has been found to involve micro-vascular shutdown, DNA fragmentation, and generic immune stimulation^2^,^3^.

ZnO nanoparticles are the auspicious material for optoelectronics devices and laser applications because of their large binding energy (60 meV) at room temperatures. In addition, ZnO nanomaterials are popular because of their biocompatibility. They embody a high quantum yield and size-dependent, tunable emission spectrum over a wide range of wavelengths^4^,^5^. Previously, several metal oxide nanoparticles have been employed in various malignant cellular models. The pharmacokinetics and biodistribution of employed nanoparticles are studied by applying various techniques. It was shown that TiO_2_ labelled with ZnPc accumulates in mitochondria and when exposed to 597–752 nm, significant photo-toxicity was reported^6^.

ZnO nanoparticles in an aqueous suspension produce singlet oxygen and hydroxyl radicals and irradiation with a blue light can enhance the oxy-radical production^7^. The ability of cancer cells to become resistant to a wide range of anticancer drugs remains a significant obstacle to successful treatment^8^. The efficient drug delivery of anti-multidrug resistant agents would have a tremendous impact in the field of cancer therapy. This study presents data demonstrating that multilayer zinc oxide nanowires that are conjugated with protoporphyrin1X (Pp1X) will emit white light after irradiation using UV light (λ = 240 nm). This phenomenon results in excitation of PpIX and liberation of reactive oxygen species, e.g., production of singlet oxygen/free radical formation, which leads to cell death. The novelty of this work is the use of multilayer ZnO nanomaterials (NMs) as a “tool” to stimulate a photochemical reaction in the targeted/tumorous site in the cell. In a previous report, there was no strong evidence that ROS kills the cell^9^.

## Results and Discussion

Predominant changes were observed when multilayer ZnO NWs grown using the femtotip probe were used for intracellular drug delivery. The idea of the multilayer femtotip was employed for the deep emission light threshold, which can allow for photochemical reactions and reactive oxygen species (ROS) liberation with the influence of molecular oxygen and PpIX within the tumour site and the surrounding tissue. Effort has been made to overcome the deficiency in drug availability at the targeted site at a threshold dose of light and the imminent challenges in PDT. Our experimental strategy allowed us to compare previously published work with current experimental outcomes. Thus, we were compelled to demonstrate the scientific reasoning of the current experimental model. In prior reported data, a lack of drug availability at the cancerous site and a non-significant dosage of light were observed. The morphology and structure of the ZnO NWs on the capillary tip were visualized using a scanning electron microscope (Fig. 1(a)). The ZnO thin film grown on the femtotip capillary is depicted in Fig. 1(b), and multilayer ZnO NWs were approximately 1.5 μm in length and 100–120 nm in diameter (Fig. 1(c) and (d)). The complete XRD analysis (Fig. 2) describes the wurtzite structure of ZnO. First, three peaks corresponded to a pure ZnO material and the fourth peak was relevant to Ag nanomaterials. Deep emission photodynamic therapy was achieved. A single layer of Ag nano thin-film deposit on a borosilicate material and continuously homogeneous layers of ZnO thin film and ZnO NWs were fabricated for bullet tool therapy. The ZnO nanowire showed a peak at approximately 33.38° corresponding to the (0002) spacing of the wurtzite structure of ZnO; the occurrence of this peak indicates preferential alignment in the c-axis direction. Two other XRD peaks were observed at approximately 34.36° and 38.04°; these peaks indicate vertically grown ZnO (0002) nanowires and deposited Ag (111), respectively. ZnO nanowires were grown on pure Ag (111), then the lattice mismatch was evaluated as 78.49%. This result means that ZnO (002) on Ag (111) has a compressive stress and must exhibit a higher XRD peak position than pure ZnO (002). When a capillary with ZnO NMs on the tip was inserted into the melanoma cells by saving its nucleus as depicted in Fig. 3(a), the cells shrunk (Fig. 3(b)). However, the shape of the cell was maintained. Furthermore, when the tip with ZnO NWs + PpIX was inserted inside the nucleus, the cell began to shrink immediately and a significant increase in fluorescence was observed even after 30 seconds, as shown in Fig. 3(c) and (d). In previously reported data, when the photo sensitizer aminolevulinic acid (ALA) was applied to a tumour, the cells accumulated protoporphyrin 1X via the heme biosynthesis pathway^10^,^11^. The protoporphyrin 1X level has been found to be greater in tumour cells because of the skin barrier^12^,^13^ and enzymatic differences^14^ as compared with normal skin. By directly inserting the ZnO NWs-containing tip inside the cell, we overcame the hindrances from Pp1X as well as other efficient photosensitizer diffusion through the cell membrane. The nano revolution has overcome the limitation of drug pharmacokinetics uptake at the oncogenic site and has provided an appropriate opportunity in the field of nanomedicine via innovation of the improved penetrability and retention (IPR) influence. Because of the severe condition of malignancy as well as local infectious diseases, nanoparticle-targeted cancer therapy has captured the attention of many investigators and oncologists, and plentiful research efforts have been made in this field. Furthermore, there has been much advancement in the last decade, e.g., nanoparticle-based targeted cancer therapy has emerged as a prevailing treatment strategy for numerous severe diseases, which is a basic need in this current era^15^. As long as advancements in traditional therapies (associated with conventional nanoparticle formulations) occur, and science shifts towards non-traditional geometries of nanoparticles for improved vascular dynamics or functionalization and more rational ways of drug delivery to overcome multidrug resistance (MDR)/drug hindrance at desired sites, specific impediments will arise which may impede clinical interpretation^15^. This may not only result in appreciation of the induction of novel therapy systems but will also bring forward nanoparticle-based reliable drug delivery formulations with more practical treatment of several local and cancerous diseases. Although more developments in the field of targeted cancer therapy (induction of novel chemical entities, conventional nanoparticles, launching of new therapies) for premalignant and malignant treatment purposes have been made in the last century, there are numerous remaining challenges like insignificant and nonspecific drug distribution, inadequate accumulation of therapeutics in the targeted site, and severe side effects caused by the unnecessary uptake of photosensitizers in healthy tissues. In cancer patients, malignant transformation of cells triggers activation of innate and adaptive immune responses, which play a critical role in controlling the growth of tumours, and are known to produce a broad variety of immunosuppressive factors in the microenvironment^16^. Tumour-induced immune cell dysfunction of adaptive and innate immunity can be observed in monocyte macrophages, natural killer cells, dendritic cells, B cells, and T cells, promoting tumours to escape from the host immune control^17^,^18^. Recent insights into immunotherapy for cancer are aimed at the anti-tumour effector cells and T cells. Prominent immunosuppression mediated by regulatory T cells plays a dynamic role in malignant lesions for assessment of tumour immunity. On the basis of this analogy, many novel treatment therapies like antibodies against superficial molecules have been established. However, few of these schemes have clinical effectiveness in melanoma patients and *in vivo* models^19^.

For the third step in the experimental scheme, melanoma cells were cultured in suitable conditions (10% FBS, 5% CO_2_, 37 °C, and in the presence of penicillin and streptomycin). These cells were exposed to various concentrations of ZnO NWs, PpIX, and a complex of ZnO NWs + PpIX under UV exposure. Unexpected results were found when melanoma cells were exposed to the same concentration (500 μg/mL) of ZnO NWs and PpIX, and different PDT results were observed in melanoma cells as depicted in Fig. 4(a). Melanoma cells exposed to 500 μg/mL of ZnO NWs are shown in Fig. 4(b). Figure 4(c) and (d) show the labelled melanoma with 500 μg/mL of PpIX and ZnO NWs + PpIX under UV exposure. Melanoma cells appear as ‘shrunken’ cells with enormous blebs at the plasma membrane with an ill-defined structure (Fig. 4(d)). In addition, ZnO NWs alone did not evoke significant cell toxicity at concentrations below 100 μg/mL in melanoma and human foreskin fibroblasts in the absence of any light irradiation, and the results resemble those of previous studies^12^. Next, we investigated the cytotoxic effects of both ZnO NWs alone and ZnO conjugated with Pp1X in foreskin fibroblasts. After 24 h incubation in the dark, we found that ZnO NWs conjugated to PpIX are more toxic at concentrations below 100 μg/mL in contrast with ZnO NWs alone in melanoma cells. Figure 5(a) shows the controlled form of foreskin fibroblasts. Figure 5(b) shows the cytotoxic behaviour of ZnO NWs (500 μg/mL concentration). Similarly, Fig. 5(c) shows the ill-defined shape of foreskin fibroblasts when exposed to PpIX, and a snapshot (Fig. 5(d)) illustrates the cytotoxic response of ZnO NWs + PpIX under UV exposure. The non-fluorescent compound carboxy-H2DCFDA (2,7-dichloro-dihydrofluoresce in diacetate acetylester) was used to detect the intracellular ROS liberation. It easily invades the cell membrane and is not fluorescent. Inside the cell, the acetate groups are hydrolysed. In this way, the substance becomes less prone to leave the cell. This new substance is not fluorescent, but it can react with ROS and produce a highly fluorescent product, as ROS will oxidize this new substance. The resulting product is fluorescent. This product’s fluorescence increases in the presence of ROS. Melanoma cells (skin cancerous model) were incubated with ZnO NWs (concentration 500 μ/mL), and after 21 h cells were examined via microscopy after excitement with a blue laser (488 nm). When the exposed cells were analysed using a conventional microscope, very intense green fluorescence was observed after exposure to ZnO NWs, but very low intensity green fluorescence was detected in the case of foreskin fibroblasts (model), and is shown as having the same algorithmic parameters of the experimental scheme. When ZnO NWs conjugated to Pp1X were exposed to melanoma, the mixture/contrast of red and green fluorescence was recorded, when excited by green light (556 nm).

The fluorescence spectrum demonstrated five peaks of white light. The first, second, and third emission peaks were at 315 nm, 400 nm, and 470 nm, respectively, and the last two peaks were at 555 nm and 625 nm, and were ascribed to a complex of monomers, oligomers, and dimers. The fifth peak in this pattern (data shown in Fig. 6) is very important, because PpIX needs 625 nm for the excitation mechanism. The relevant peak provides the threshold for liberation of photochemical reactions, which lead to ROS, resulting in the cell killing mechanism. A number of scholars have claimed that ZnO is bio-safe and biocompatible^20^, but we have found that bare ZnO NWs and those conjugated to Pp1X exhibit considerable cell toxicity to fibroblasts and melanoma cells when incubated together for 24 h. Because of the high aspect ratio, ZnO nanowires can be used for tumour-selective delivery of chemotherapeutic agents. For verification, mitochondria of treated melanoma were stained with Mito Tracker Red to visualize the mitochondrial membrane potential, as shown in Fig. 7(a–d). The figure depicts microscopic images of treatment provoking heavy damage to the cell including the mitochondria, via rapid fluorescence increase after 20 minutes of UV irradiation. These results were confirmed by applying ROS analysis and staining cells with Mito Tracker Red CMXRos (200 nM, 37 OC Invitrogen). It was observed that after 25 hours of cell treatment, loss in mitochondrial membrane potential was observed in addition to ROS production. The same trend was seen in foreskin fibroblasts.

Figure 8 describes the PDT. The basic novelty was that deep emission PDT was established for the first time. The first layer of the borosilicate silver-coated femtotip capillary was coated with a ZnO thin film within the nano-range and the second and final layer of ZnO NWs were grown on the ZnO thin film grown on the silver-coated femtotip capillary. In the second step, the multilayer ZnO NMs-grown femtotip was conjugated with 600 μg/mL working solution of PpIX. Then, manual insertion of this bullet tool was performed, saving the nucleus and mitochondria. During insertion of the femtotip into the melanoma as well as the foreskin fibroblast, 20 J/cm^2^ of UV light was irradiated. This UV light was employed for excitation of ZnO NWS and ZnO thin film; as a result, we achieved the threshold value of red light from the broadband emission spectrum of white light. PpIX, in the presence of the threshold light and molecular oxygen in the neighbouring territory of the targeted site, was able to produce a significant quantity of photochemical reactions/ROS liberation, leading to the loss of the mitochondrial membrane and finally resulting in cell death. Figure 8 shows the scientific manifesto of PDT. Before this experiment, the scientific model based on a single layer of PDT was reported but deep emission PDT and the concept of multilayer ZnO NMs are novel in this current experiment. Figure 9 shows the PDT protocol flow chart.

To study the cytotoxic mechanism of both ZnO NWs alone and ZnO NWs conjugated with PpIX against melanoma and foreskin fibroblast cells, the cells were exposed to ZnO NWs (0–600 μg/mL), Pp1X alone, and ZnO NWs conjugated with PpIX in the dark as well as under UV light. Finally, cell viability was assessed using the MTT assay after 21 hours. Unexpectedly, no significant apoptotic/necrotic effects were observed in the foreskin fibroblasts even at concentrations up to 500 μg/mL of PpIX. Healthy tissues have a stronger immune system compared with malignant tissues. Numerous scientific phenomena are responsible for the failure of tumour antigen T cell feedback controls resulting in immune collapse. A series of complex chemical changes are involved in somatic genetic alterations (from benign lesions to metastases phases), but the actual mechanisms from the primary to final stages of metastases are under debate. To further clarify these mechanisms, studies have been performed using normal as well as malignant skin cellular models^21^. Melissa Q McCreery revealed that lymph nodes are the main factor affecting metastasis after a linear model experiment was carried out on primary stage lung and liver cancer using mice^21^. Interesting results were observed when the experimental study was employed on primary stage skin cancer and metastasis using a mouse model^22^. Reliable therapeutically technique for evaluation of dissemination or metastatic clinical setting^21^.

When comparing the cytotoxicity results, it was found that foreskin fibroblasts are more resistant than melanoma cells. Working solution of ZnO NWs (600 μg/mL), PpIX, and ZnO NWs + PpIX under UV irradiation and in the absence of UV were investigated. Cytotoxicity and phototoxicity were examined in the presence and absence of UV exposure in the foreskin fibroblasts as well as melanoma cells, as shown in Fig. 10. Significant loss in cell viability in melanoma cells was observed after exposure to 600 μg/mL of ZnO NWs + PpIX under 20 J/cm^2^ UV light. The percent loss in cell viability reached 70%, and only 30% of cells were living, as assessed by MTT assay, but under the same experimental conditions the loss of foreskin fibroblast viability was 50%. The difference in toxic concentrations between fibroblasts and melanoma might be a result of healthy tissues having strong immune properties as compared to malignant tissues and different rates of cell proliferation, which were 5-fold greater in melanoma cells compared with fibroblasts. The toxicity of a nanomaterial depends upon the chemical and phototoxicity caused by the discharge of toxic ions and formation of reactive oxygen species. Moreover, the shape and size of the NWs might induce mechanical trauma at the plasma membrane^23^. Similar results were obtained using ZnO nanoparticles^24^. In short, cytotoxicity as well as phototoxicity is dependent on size, morphology, concentration, and addition of the laser (wavelength of light ≈240 nm for liver tissue and 630 nm for other cells). ZnO NWs as well as ZnO nanomaterials are safe and biocompatible up to a certain limit and can be used as drug delivery vehicles. Above the threshold dose, its concentration is toxic even in normal tissues/cells.

Equation 1 describes the empirical model for the experimentally obtained data of ZnO melanoma ROS. The unknown variables in equation 1 are extracted via the least square error method and are listed in Table 1. It is noted that the magnitude (*a*_*i*_) of the first sine term with lowest frequency (*b*_*i*_) is highest compared to other high frequency sine terms. The magnitude of the other sine terms decreases with increasing frequency. Phases (*c*_*i*_) of the sine terms are adjusted to have the least mean square error in the model when compared with the experimental data.



Where  unknown constants are extracted through the method of least square errors and listed in Table 1, x represents ZnO NMs and its complex concentration, μg/ml.

Other experimental data for fibroblasts, melanoma cells, PpIX with melanoma cells, PpIX with fibroblasts, and ZnO with fibroblasts were also weighted with appropriate factors and projected in the empirical model of equation 1. These weighting factors (*K*_*i*_) are also extracted from the method of least square error and are listed in equations 2,3,4,5,6. Figure 11 shows that the weighted factor experimental data is close to the empirical model of equation 1. In order to show the accuracy of the proposed model, P-value analysis is performed for each experimental data point against the empirical model of equation 1. All the P-vales are listed in Table 2.











It is therefore concluded that our experimental results regarding ZnO melanoma ROS, fibroblasts, melanoma-PpIX, PpIX-fibroblast, and ZnO-fibroblast are in good agreement with the model of ZnO for melanoma.

## Conclusion

In conclusion, we observed that multilayer ZnO NWs are useful for deep emission photodynamic therapy (DEPDT). Femtotip tools can be used as a magic bullet for drug delivery by achieving the light threshold necessary for significant ROS production, leading to cell killing effects. Multilayer ZnO NWs conjugated with PpIX under UV exposure were employed in human melanoma cells (FM55P) and human foreskin fibroblasts cells (AG01518) as models for toxicity evaluation by applying the microinjection drug delivery technique. Multilayer ZnO NWs provide a favourable amount of PpIX during conjugation and the necessary light threshold when excited with UV light for significant photochemical reactions causing loss in mitochondrial membrane potential and significant loss in cell viability. Significant photochemical reaction presence was investigated in the bioavailability of the significant PpIX light threshold under UV irradiation. It was proven that normal skin cells are more resistant than skin melanoma. Results were confirmed by applying various advanced techniques. The mathematical model verifies the experimental model. We denounce the biosafety and biocompatibility of ZnO NMs, with their cell killing effects due to their shape, size, and morphology. Currently, the bio-safety of ZnO NWs might be questionable. These potent nanoparticles may be capable of improving targeted drug delivery and site-specific deep emission photodynamic therapy. Their use might result in a viable treatment for several invasive diseases. Currently, the field of nanomedicine is extending beyond the confines of traditional experimental schemes (e.g., traditional geometries, sizes, or chemistries), and there are formidable challenges associated with this strategy. Advancements in therapies will pave the way for more rational designs for targeted drug delivery techniques.

## Materials and Methods

### Synthesis and morphological analysis of grown multilayer ZnO NMs on femtotip glass borosilicate capillary

The main emphasis was on the fabrication of homogeneous multilayered ZnO NMs on the tip of a silver-coated borosilicate femtotip with capillary geometry. An extremely sharp tip and multilayered grown zinc oxide nanomaterials (ZnO NMs) for deep emission photodynamic therapy (DEPDT) were introduced for the first time. The basic idea is that the optimal values of the drug, light, and molecular oxygen are responsible for reliable and effective photodynamic therapy (PDT). In this experimental strategy, our femtotip tool will be able to overcome the deficiency of drug availability as well as light threshold dosage (from emission of broadband light when ZnO NMs are excited with UV light). Development of a safe intracellular therapy device is the novelty of the current experimental scheme. Properties of bending and gentle penetration in the cell membrane were included as features of the femtotip tool.

An innovative and unique strategy was implemented for deep emission photodynamic therapy (DEPDT) in foreskin fibroblasts as well as skin melanoma cells. The borosilicate capillary (sterile Femtotip ^®^ II Eppendorf) with a special probe that had an internal diameter less than 0.5 μm (external diameter 0.7 μm) was employed and the inserted length was approximate 1 mm. Prior to growth of multilayer ZnO NMs, borosilicate glass femtotip capillaries were prepared in subsequent steps. Thin films of silver and chromium having thicknesses of 20 nm and 120 nm, respectively, were uniformly placed onto the superficial surface of the femtotip capillary tips. On the silver-coated glass borosilicate capillary tip, hexagonal multilayer shapes of crystals of a monolayer of ZnO thin film were fabricated in the first step, and after etching/trimming the spare ZnO thin film, ZnO NWs were grown in the appropriate environment^9^,^25^,^26^. For the synthesis protocol, the following steps were implemented. (NH_4_)_2_CO_3_, Zn(NO_3_)_2_.6H_2_O, and NaOH were thawed in distilled water to prepare a 1.0 M (NH_4_)CO_3_ solution, 1.0 M Zn(NO_3_).6H_2_O solution, and 1.0 M NaOH solution, correspondingly. A 1.0 M Zn (NO_3_)_6_H_2_O solution (100 mL) was dropped gently into 250 mL of a (NH_4_)_2_CO_3_ solution with vigorous stirring to attain a precipitate. The mixture was strained and constantly rinsed with deionized water to eliminate the remaining reactants. Next, it was dissolved in 300 mL of deionized water for 30 minutes. A 1.0 M NaOH solution was added to this dispersion to adjust the pH to 9.2. This suspension was transferred to a Teflon-lined stainless autoclave with an optimal value of 500 mL and exposed to 200 °C for four hours. After completion of the reaction, the finalized form of powder (white) product was filtered via suction and dehydrated in a vacuum at approximately 100 °C. The ZnO thin film as well as ZnO NWs were attained by calcining the powder form at 460 °C for two and half hours.

A multilayer ZnO NMs-grown femtotip was conjugated to a protoporphyrin 1X (Pp1X) layer via a manual process, as described^9^. For toxicity measurement, insertion of a laboratory-made femtotip tool bare monolayer ZnO thin film, multilayer ZnO NWs grown tips, and multilayer-grown ZnO thin film in the inner surface and ZnO NWs in the upper/outer surface (called homogenous multilayer grown ZnO NMs) conjugated with PPIX into FM55P and AG01518 were also included in the on-going experimental strategy. The concentration of PpIX was 80 mg/mL (pH 5.5 or 7.0; Sigma Aldrich, Sichuan, Chengdu China) dissolved in N-dimethyl formaldehyde (Sigma Aldrich, Sichuan, Chengdu China). After conjugation of the working solution PpIX with the multilayer grown ZnO NWs femtotip, fluorescence emission spectroscopy was employed for confirmation of the perfect complex of ZnO NWs with PpIX.

Free-standing drug delivery ZnO nanowires (ZnO NWs) were synthesized via a chemical aqueous method under an optimized environment. The desired morphology of the ZnO NWs was acquired by repetition of sample growth. Free-standing zinc oxide NWs were dispersed in distilled water via a vortex and ultra-sonication process for 25 minutes to form a homogenous stock solution of 10 mg/mL, and the working solution was then prepared using different concentrations (0.05–600 μg/mL). The same procedure was used in the conjugation of ZnO NWs with PpIX working solutions. Biotoxicity of ZnO NWs alone, PpIX alone, and ZnO NWs conjugated with Pp1X solutions were tested separately by applying the MTT assay. Intracellular measurements were performed on the stage of a Carl Zeiss (Carl Zeiss, Meditec AG, Tokyo Japan) inverted microscope, using a mechanical manipulator (Eppendorf) to fix the ZnO NWs.

Finally, the statistical data was collected from the experimental results and analysed with the least square errors method. The weighted sinusoidal representation for all the experiments was best suited and generated the least mean square error when compared to the original data. The trend in all the experiments remained the same, enabling a single mathematical model to represent all the experiments with a single equation having different weights, as discussed in Section 3.

### Cells and culture conditions

Human melanoma cells (FM55P) were subcultured in tissue culture flasks with a diameter of 25 cm^2^ with minimum essential media (MEM) with Hanks salts, foetal bovine serum (10%), 100 U/mL penicillin, 100 μg/mL streptomycin, 100 μg/mL fungizone, and 2 mM L-glutamate. Human foreskin fibroblasts (AG01518) were seeded in 24 well plates in Eagle’s modified minimum essential medium (EMEM) containing 10% foetal bovine serum, 2 mM glutamine, 45 U/mL penicillin-G, and 45 mg/mL streptomycin. Both cultured form of cells were maintained and incubated at 37 °C in humidified air with 5% CO_2_ and were subcultured three times a week. Prior to experimentation, cells were trypsinised and seeded at concentrations of 30000 cells/cm^2^ for melanoma cells and 25000 cells/cm^2^ for fibroblasts^27^,^28^.

### Experimental scheme

Human melanoma cells (FM55P) and human foreskin fibroblasts (AG01518) were seeded in glass petri dishes. In the first step, the ZnO NWs multilayer grown femtotip probe was inserted manually into human melanoma cells (FM55P) and human foreskin fibroblasts (AG01518), respectively, avoiding the nucleus. In the second step, a PpIX-conjugated ZnO NWs multilayer grown femtotip tool was inserted in the presence and absence of UV exposure. Later, cells were cultured in 96 well plates, and biotoxicity of ZnO NWs alone, PpIX alone, and the ZnO NWs + PpIX complex was tested in normal and cancerous skin cell models under UV exposure. Four rows in each column were specified for each sample, and each sample was employed five times in the experiment. Data were evaluated by applying various confirmatory tests and analysed statistically.

### Analysis of mitochondrial membrane potential

To examine the actual cell killing effects, after experimentation, the above mentioned cells were labelled with Mito Tracker Red CMXRos (200 nM, 37 °C, Invitrogen) for 40 minutes to determine the actual condition of mitochondrial membrane potential. All cultured cells were maintained in serum free media. At the end of the experiment, fresh medium was added to the labelled cells and snapshots were captured after examination with a Carl Zeiss (Carl Zeiss, Meditec AG, Tokyo Japan) inverted microscope using a Nikon photomicroscope.

### Cell viability

Human melanoma cells (FM55P) and human foreskin fibroblasts cells (AG01518) were cultured in 24-well plates and exposed to 0.05–600 μg/mL of ZnO NWs, 500 μL of PpIX, and 500 μL ZnO NWs conjugated with PpIX. Each concentration was assigned to four wells in each row and the fifth and sixth wells in each row were considered control wells in 24 well plates. Control cells were incubated either with serum or without serum. Cells were incubated in humidified air with 5% CO_2_ at 37 °C for 24 h. For cell morphological analysis, microscopy was performed. Images of treated and control cells were captured. Cell viability was tested using the MTT assay. The MTT assay was performed via the addition of 2-(4,5-dimethyl-2-thiazolyl)-3,5-diphenyl-bromide (0.25 mg/mL in phosphate buffer saline) to the cultured plate, and cells were incubated for 3 h at 37 °C in humidified air with 5% CO_2_. The sample plates were then dried, and formazan agent was thawed in DMSO for further steps. The cell absorbance was examined at 570 nm (available Optical Filter 340 nm, 414 nm, 492 nm, 570 nm, 595 nm 630 nm, and 650 nm) using a microwell plate reader (Multiskan FC R, Microplate Photometer Thermo Fisher SCIENTIFIC).

### Reactive oxygen species (ROS) detection

Intracellular reactive oxygen species (ROS) liberation was tested by labelling the non-fluorescent complex CM- H2DCFDA (2, 7-dichlorodihydrofluoresce in diacetate acetyl ester; Invitrogen Co., USA). This compound enters into the cell membrane by endocytosis and undergoes deacetylation by esterase, creating the non-fluorescent CM-H2DCF. Cells were cultured in a plastic 96-well plate and labelled with different concentrations of ZnO NWs, ZnO NWs-conjugated PpIX, and ZnO NWs with ALA in humidified air with 5% CO_2_ at 37 °C for 12 h. The cells were washed gently once with Dulbecco’s modified Eagle’s medium (DMEM).

Cells encumbered with 100 μL of 5 μM CMH2DCFDA were maintained for 30 minutes at 37 °C and sheltered from light exposure. Thereafter, the cells were exposed to 20 J/cm^2^ of UV light for 2 minutes and then were examined for ROS via fluorescence using a calibrated microwell plate reader (Multiskan FC ^®^, Microplate Photometer Thermo Fisher SCIENTIFIC). Cells were also seeded in glass petri dishes, labelled, and irradiated per the recommended procedure. They were then excited via exposure to blue light (488 nm), and images were captured under an inverted fluorescence microscope with a digital camera^29^.

### Mathematical Model

As shown in Fig. 11 and Table 3, there were six different sets of experiments with entirely different ranges of values for reactive oxygen species (ROS) fluorescence (a.u). Therefore, six different expressions were required in order to model these experiments. However, this paper proposes a single model for all these experiments. A simple empirical model based on weighted sinusoidal functions is proposed for experimentally obtained values of ZnO melanoma ROS. The weighted sinusoidal model guaranties the regeneration of almost any function from its constituent frequencies. The reason for selecting weighted sinusoidal functions is that the experimental data does not follow any monotonic linear or exponential trend. Other candidate functions such as bi-harmonic or thin-plate spline are complex and rarely used in extraction of simple empirical models. After selection of the weighted sinusoidal function as a basic function to generate the model, the method of least square error was applied to obtain a 95% confidence interval. It was observed that only three sinusoidal terms were sufficient to generate the model with 95% accuracy for this data. Utilizing more sinusoidal terms in the model will improve the accuracy at the cost of more coefficients. A simple model is required with fewer numbers of coefficients for the 95% confidence interval, so there is no need for adding any additional terms. All other experiments are projected on the ZnO melanoma ROS model with different weights. These weights are also extracted using the method of least square error. Taking any other weights will lead to more mean square error in the model.

## Additional Information

**How to cite this article:** Fakhar-e-Alam, M. *et al*. Empirical Modeling of Physiochemical Immune Response of Multilayer Zinc Oxide Nanomaterials under UV Exposure to Melanoma and Foreskin Fibroblast. *Sci. Rep.* **7**, 46603; doi: 10.1038/srep46603 (2017).

**Publisher's note:** Springer Nature remains neutral with regard to jurisdictional claims in published maps and institutional affiliations.

## Figures and Tables

**Figure 1:** Scanning electron micrograph of (**a**) A silver-coated capillary tip as PDT device. (**b**) Homogeneous layer grown on ZnO thin film model on silver coated femtotip capillary. (**c**) SEM image of ZnO nanowires on the silver-coated capillary tip having a scale range of 1 μm with the inset showing the hexagonal ZnO nanowires. (**d**) SEM images magnified from a selected area of ZnO NWs grown on a femtotip capillary having a scale range of 1 μm for deep emission photodynamic therapy.

**Figure 2:** XRD analysis of silver-coated ZnO fabricated capillary tip as a PDT device.

**Figure 3:** Microscopic view of (**a**) phase contrast image of ZnO nanowires capillary conjugated to PpIX and inserted into a fibroblast. (b) Reflex image of ZnO nanowires with capillary conjugated to PpIX just after insertion. (c) ZnO nanowire capillary tip near a single stained fibroblast. (d) Foreskin fibroblasts stained with Mito Tracker Red to visualize mitochondrial membrane potential.

**Figure 4:** Cytotoxicity of melanoma cells. (**a**) Control melanoma cells. (**b**) Melanoma cells exposed to 200 μg/mL of ZnO. (**c**) Melanoma cells exposed to ZnO-grown, 60 μg/mL PpIX-doped femtotip capillary. (**d**) Melanoma cells exposed to 250 μg/mL of ALA.

**Figure 5:** Cytotoxicity of human foreskin fibroblasts. (**a**) Control fibroblast. (**b**) Fibroblasts exposed to 10 μg/mL ZnO + Pp1X. (**c**) Human fibroblasts treated with Pp1X (250 μg/mL). (**d**) Human fibroblast exposed to 250 μg/mL of ZnO NWs + ALA.

**Figure 6:** Florescence (Fl) Emission spectra of multilayer ZnO NWs conjugated with PpIX. The spectra captured by applying 240 nm light as an excitation source from a PTI- Fluorescence system.

**Figure 7:** Microscopic images of (**a**) control melanoma cells with serum (FM55P), (**b**) insertion of femtotip capillary into melanoma cells, (**c**) insertion of femtotip capillary into melanoma cells under UV exposure, (**d**) microscopy of melanoma cells stained with Mito Tracker Red and the ZnO nanowires tip inside a cell after UV exposure.

**Figure 8:** Science of photodynamic therapy.

**Figure 9:** Complete photodynamic therapy (PDT) procedure flow chart.

**Figure 10:** Percent cell viability loss in melanoma before and after irradiation with UV light (having 240 nm of light wavelength, 20 J/cm^2^ threshold dose).

**Figure 11:** Reactive oxygen species (ROS) mathematical model developed from experimental model using normal skin and skin melanoma.

**Table 1:** Values of different constants, extracted from the method of least square error, for equations 1, 2, 3, 4, 5, 6.

P	V	P	V	P	V	P	V
*a*_1_	17170	*a*_2_	127.7	*a*_3_	59.2	*b*_1_	0.0006374
*b*_2_	0.0938	*b*_3_	0.2098	*c*_1_	0.03405	*c*_2_	2.003
*c*_3_	−1.308	*K*_1_	0.973684211	*K*_2_	0.419858156	*K*_3_	0.967320261
*K*_4_	1.947368421	*K*_5_	2				

P = Parameter V = Value of Parameter.

**Table 2:** P-values of ZnO melanoma ROS Model compared to the other experimental data.

		P-value
1	ZnO Melanoma ROS	0.003
2	Fibroblast*K_1_	0.0025
3	Melanoma*K_2_	0.0226
4	PpIX Melanoma*K_3_	0.0058
5	PpIX Fibroblast*K_4_	0.032
6	ZnO Fibroblast*K_5_	0.047

**Table 3:** Values of ROS fluorescence (a.u.) of different experiments with changing ZnO NMs and its complex concentration.

ZnO NMs, and its complex concentration	Fibroblast	Melanoma	PpIX data for Melanoma ROS	PpIX data in Fibroblast ROS	ZnO Data for Fibroblast ROS	ZnO Data for Melanoma ROS
10	750	1600	720	370	350	650
20	800	1800	810	376	360	750
30	820	1900	810	368	355	760
40	750	2000	730	345	335	680
50	1150	2550	1100	545	530	1050
60	1300	3000	1190	570	560	1150
70	1480	3450	1410	680	660	1350
80	1505	3500	1510	745	730	1450
90	1520	3525	1530	760	740	1480
